# Automated Prediction of Employee Attrition Using Ensemble Model Based on Machine Learning Algorithms

**DOI:** 10.1155/2022/7728668

**Published:** 2022-06-26

**Authors:** Fahad Kamal Alsheref, Ibrahim Eldesouky Fattoh, Waleed M.Ead

**Affiliations:** ^1^Information Systems Department, Faculty of Computers and Artificial Intelligence, Beni-Suef University, Beni-Suef, Egypt; ^2^Computer Science Department, Faculty of Computers and Artificial Intelligence, Beni-Suef University, Beni-Suef, Egypt

## Abstract

Competent employees are a rare commodity for great companies. The problem of maintaining good employees with experience threatens the owners of companies. The issue of employee attrition can cost employers a lot as it takes a lot to compensate for their expertise and efficiency. For this reason, in this research, we present an automated model that can predict employee attrition based on different predictive analytical techniques. These techniques have been applied with different pipeline architectures to select the best champion model. Also, an autotuning approach has been implemented to calculate the best combination of hyper parameters to build the champion model. Finally, we propose an ensemble model for selecting the most efficient model subject to different assessments measures. The results of the proposed model show that no model up until now could be considered ideal and perfect for each case of business context. Yet, our chosen model was pretty much optimal as per our requirements and adequately satisfied the intended goal.

## 1. Introduction

Currently, machine learning and data mining are considered the most effective and active research areas. Different data mining techniques are used in classification, clustering, and prediction [1, 2]. Because of the importance of data mining and machine learning, many other methods are applied in different fields, such as education, healthcare, banking, security systems, mobile game industry, and human resource management [3, 4]. Employee attrition is a drop in the number of workers of an organization, where the employees have left the business voluntarily or retired. In any organization, highly efficient employees are considered the most valuable asset [5]. Retaining the most marketable or high-performance employees is a big challenge in many organizations. The problem of employee turnover (attrition) has gained popularity in many organizations because of its adverse effects on various subjects ranging from organizational performance and efficiency to disturbances in projects' progress and long-term growth strategies [6]. In fact, this problem adds new spending on organizations to spend more on human capital, recruitment, preparation, and development for the new staff [7].

For the reasons given above, organizations need to predict the level of attrition and keep their employees through more reasonable company policies and regulatory environments. The current research would help most companies to know the level of satisfaction of their employees and obtain some valuable information, which would help control the attrition rate. In the current research, a machine-learning model founded on artificial neural networks and support vector machines was proposed to predict employee attrition for assisting organizations to control the attrition rate.  Section 2 of the paper offers literature review about employee attrition and other prediction models using machine-learning methods.  Section 3 will designate different machine learning algorithms used in the projected model. The used data set and investigational results of this study will be discoursed in Section 4. Lastly, the conclusion and future work will be offered in Section 5.

The main contribution of this work has many objectives. On the one hand, it is addressing the challenge of employee attrition problem. On the other hand, it is addressing different machine learning techniques that create an ROI to help the enterprises understand the real causes of why the employees are churned. Moreover, the proposed model will be used as an alert to the enterprise's human resource decision makers to prevent their employees from being churned. In addition, it is presenting new outcomes supporting or opposing the current study and the other literature available on this particular domain.

## 2. Related Work

In this section, we present a literature survey on some employee attrition models implemented in many pieces of research. In their study, Sisodia et al. [5] built a prediction model for employee churn rate. They used five machine learning algorithms, such as linear support vector machine and C5. Decision tree, k-nearest neighbor, Naïve Bayes classifier, and random forest outperformed all other classifiers. Alao and Adeyemo [7] generated five different decision tree models and two rule sets. The generated output from both is used to develop a prediction model for predicting new cases of employee attrition. Another study to evaluate different machine learning algorithms in predicting employee attrition was presented by Zhao et al. [8]. Ten different algorithms were applied in that study on three different datasets. The datasets represent organizations of various sizes, ranging from small-, medium-, and large-sized employee populations. The study concluded that no algorithm outperforms the others in the small dataset. In the medium dataset, the extreme gradient boosting trees result in greater accuracy, while in the large dataset, the gradient boosting trees were the recommended algorithm. A prediction model for prioritizing the features with a high impact on employee attrition and its causes is presented in the study of Yadav et al. [9]. They applied many machine learning techniques, and the decision tree brought about the highest accuracy in their experiment on experienced employee data. In another study by Khare et al. [10], the logistics regression method was proposed to develop a risk equation for predicting employee attrition based on separated and existing employees' demographic data. Far ahead, the same equation was applied for estimating attrition risk with the existing positioned workers. The cluster with higher chances was defined to discover the reasons and help build a strategy for minimizing risk. In another employee attrition model presented in Alduayj and Rajpoot's [11] study based on machine learning, three experiments were applied, and in each one, three algorithms were used. The first experiment was on the original data, which was imbalanced. In this experiment, the SVM algorithm reported the best F1 score value. They provided an adaptive synthetic sampling method in the second experiment to overcome the class imbalance problem. It was noticed in that experiment that the performance of all methods enhanced. In the last experiment, they sampled the dataset manually, and this process led to lower performance. The study conducted by Zhu et al. [12] suggested multiple time series modeling techniques for identifying the best models to forecast employee turnover. Based on their statistical evaluation, they selected eight univariate models with acceptable R2 values, and the dynamic regression model is the top prediction model. Fallucchi et al. [13] carried out research and applied many machine learning techniques to predict the factors that may lead the employee to leave the company. The Gaussian Naïve Bayes classifier gave the best recall value that contributes to the classifier's ability to discover the positive instances. A hybrid model for customer churn forecasting was given in the study of Jamalian and Foukerdi [14]. In that model, the principal component analysis (PCA) algorithm was used in feature selection. The LOLIMOT and C5.0 algorithms were skilled with features of several sizes. The output of each classifier is merged with weighted voting, and the output of the hybrid model had a higher accuracy than individual classifiers. Also, prediction models are presented in different fields like the one presented in Arumugam's [15] study. The model is for paddy crop productivity. The author has proposed a plan for agriculture that may be of assistance to farmers.  Table 1 summarizes the machine learning algorithms used in each of the mentioned literature.

The contribution of this work is to automate and support the decision-making processes in an important and vital problem in human resource management. Furthermore, different predictive analytical techniques have been implemented with different pipeline architectures to select the best champion model to be deployed in the production environment. In addition, an autotuning technique is implemented to calculate the best combination of hyperparameters to build the champion model. Moreover, an ensemble model has been proposed to select the best efficient model subject to different assessment measures. Finally, the different proposed models were measured and compared according to different assessments and statistic measures.

## 3. Proposed Model

Building a machine learning (ML) model in a real-world environment is performed through three different phases: data, discovery, and deployment. The data phase is concerned with collecting the data, exploring the data, dividing the data, addressing the rare event issues in case of an unbalanced dataset, managing the missing values, handling extreme or unusual values, and finalizing the selection of essential features to be used by the model. The discovery phase tasks are to select an algorithm, improve the model, optimize the complexity of the model, and regularize and tune the hyperparameters of the model. Deployment phase tasks are assessing the models, comparing the ML models, and scoring the champion ML model. The primary steps for predicting the employee attrition problem in the proposed model are shown in Figure 1. Once the data is collected, it goes to the most important step in the prediction models, which is the preprocessing step. In such step, different processes, such as imputation to the missing values of the dataset and feature transformations for skewed and high kurtosis variables, are carried out. Feature transformation will help in model generalization for the new incoming data while we are scoring the model.

## 4. Material and Methods

We used a real dataset from SAS (www.sas.com) library, containing 35 variables/columns that vary from categorical and interval variables, and 1.5k rows. The following table demonstrates the data preparation setting for the concrete and interval variables.

The threshold for interval/nominal variables is shown in Table 2. In case a numeric input has extra levels compared to the interval cut-off, it will be an interval. Otherwise, it will be nominal. The maximum class level threshold is used to reject the categorical variables, if it has more class levels than the predefined threshold. If a variable has more missing values than the maximum per cent missing, then the threshold to reject missing variables will be rejected, and the partitioning ratio threshold is used for partitioning the dataset into training, testing, and validation partitions. For preliminary model fitting, the training dataset is used. Furthermore, to find the sweet spot among overfitting, underfitting, and “optimize complexity” of the model, validation data is used. Validation data fine-tunes the models built on training data and determine whether additional training is required. The test dataset is used for a closing evaluation of the model.

A stratified random sample is used as a partitioning method. Conversely, it initially splits the people into small clusters or levels according to similar features with the attrition target variable. Consequently, a graded sampling approach would assure that the members of all subgroups are involved in data assessment.

### 4.1. Proposed Model Technologies

Various machine learning algorithms were developed to learn from the data referred to as training samples. The trained model analyzes and predicts the intended class when new data are generated. In this section, we describe the ML algorithms used in prediction.

#### 4.1.1. Multilayer Perceptron Classifier (MLP)

The first paper, which introduces how neurons can work, was introduced by Warren McCulloch and mathematician Walter Pitts in 1943 [16]. A multilayered perceptron is a feedforward artificial neural network model in which the input data is mapped to a collection of suitable outputs. It has three layers, namely the input, production, and concealed layers. The input layer receives the processing signal. The processing of MLP consists of an infinite number of hidden layers between the input and output [17]. We demonstrated the backpropagation algorithm for training MLP.  Figure 2 shows a typical MLP neural network. The hidden layer is required for classifying indivisible datasets. The j^th^ output of feedforward MLP is as follows:

(1) $$\begin{array}{c} y_{j}=f\left(\sum_{i=1}^{k}W_{ij}^{2}\emptyset_{i}\left(x\right)+\;b_{j}^{2}\right., \end{array}$$

where ∅_*i*_(*x*) is the input vector, *b*_*j*_^2^ is the bias of the output neuron, and *j*(*x*) is the output of hidden neuron *i*.

(2) $$\begin{array}{c} \emptyset_{i}\left(x\right)=f\left(W_{i}^{\left(1\right)}*x\right)+b_{i}^{\left(1\right)}, \end{array}$$

where *b*_*i*_^(1)^ is the bias of hidden neuron i.

#### 4.1.2. Random Forest (RF)

A random forest is a classifier collaborative of decision trees produced by two randomization sources. Initially, all decision trees are trained on a randomly selected example of the actual data with a replacement of the identical size as the training dataset [18]. It is expected that nearly 37% of the instances in the produced bootstrap samples will be duplicated. Attribute sampling is the second randomization source used in random forests. To accomplish this, a small fraction of the input variables is chosen randomly at each node split to find the best split. The suggested value by Breiman [19] for this hyperparameter is ⌊log_2_(no_of_selected_features)+1⌋. To classify, the ensemble's final forecasting is determined by majority voting. One of the advantages of random forest is that it is hyperparameter-free, or at the very least, the default hyperparameter setting performs excellently on average [20]. In any case, other hyperparameters in the random forest that can be tuned are those that govern the decision trees' depth. Overall, in a random forest, decision trees can grow until all their leaves are genuine. The tree's growth can be constrained by demanding the fewest number of cases in each node or imposing a maximum depth before or after the split [21].

#### 4.1.3. Gradient Boosting (GB)

Gradient boosting is a regression algorithm similar to boosting [22]. The goal of gradient boosting on a given training dataset *D*={*x*_*i* _, *y*_*i*_}_1_^*N*^ is to find an approximate value, $\hat{F}$ (*x*), of the function *F*^∗^ (x), which, by minimalizing the predicted value of a particular loss function, relates instances *x* to their corresponding output values *y*, L(y, F(x)). GB generates a weighted sum of functions as an additive estimation of *F*^∗^ (*x*) as follows:

(3) $$\begin{array}{c} F_{m}\left(X\right)=F_{m-1}\left(X\right)+\rho_{m}h_{m}\left(X\right), \end{array}$$

where *ρ*_**m**_ is the weight of the m^th^ function, **h**_**m**_(**X**). These functions are the ensemble's models. The estimation is built iteratively. Firstly, a constant approximation of *F*^*∗*^ (*x*) is gained as follows:

(4) $$\begin{array}{c} F_{0}\left(x\right)=\text{argmin }\sum_{i=1}^{N}L\left(y_{i}\;,\;\alpha \right). \end{array}$$

The following models are required to minimalize.

(5) $$\begin{array}{c} \left(\rho_{m},h_{m}\left(x\right)\right)=\arg\;\min_{\rho ,h}\sum_{i=1}^{N}L\left(y_{i},F_{m-1}\left(x_{i}+\rho h\left(x_{i}\right)\right)\right.. \end{array}$$

Every *h*_m_ can be thought of as a step of the greedy step gradient descent optimization for *F∗*. To accomplish this, for every model, *h*_m_, is trained on a new dataset *D*={*x*_*i*_,  *r*_*mi*_}_*i*=1_^*N*^, with pseudoresiduals, r_mi_, obtained by the following:

(6) $$\begin{array}{c} r_{mi}={\left[\frac{\partial L\left(y_{i},F\left(x\right)\right)}{\partial F\left(x\right)}\right]}_{F\left(x\right)=F_{m-1}\left(x\right)}, \end{array}$$

where the value of *ρ*_**m**_ is calculated by resolving a line search optimization issue [21].

#### 4.1.4. Ensemble Model

Ensemble methods are the tactics to develop numerous models and merging them to produce improved outcomes. In the majority voting ensemble models, every model predicts for all test instances, and the final output prediction is the one receiving majority of the votes. Ensemble produces a new model by taking a function of posterior possibilities (for class targets) or the predicted values (for interval targets) from numerous models. The algorithm used in majority voting works as follows:

## 5. Results Discussion

As shown in Figure 1 of the projected model, different machine learning techniques have been implemented, such as gradient boosting, artificial neural networks, random forest, and ensemble models. Moreover, various performance measures have been implemented to find the most efficient machine learning techniques, such as cumulative lift, lift, accuracy, and F1 score.

Cumulative lift is evaluated by classifying all partitions in downward order by the foretold possibility of the target event P_AttritionYes, representing the expected possibility of the event “Yes” for target attrition. The data is partitioned into 20 quantiles (demideciles, with 5% of the data in each), and the quantity of events in all quantiles is calculated.  Figure 3 shows the value of cumulative lift for different algorithms in train, validation, and test partition. The cumulative lift for a specific quantile is the proportion of the number of events among each quantile up to and involving the present quantile to the number of events that will be there randomly, or consistently, the proportion of the cumulative response percentage to the baseline response percentage. The cumulative lift at depth 10 involves the top 10% of the data, the first 2 quantiles, with 10% of the events at random. Hence, cumulative lift calculations show that observing an event in quantiles is way too probable compared to randomly picking observations.

Lift measure is estimated by classifying all partitions in a downward order by the expected likelihood of the target event P_AttritionYes, representing the expected possibility of the event “Yes” for the target attrition. The data was segmented into 20 quantiles (demideciles, with 5% of the data in each), and the number of events in all quantiles are calculated. Lift is the ratio of the number of events in that quantile to the number of events that will be there randomly, or homogeneously, it is the proportion of the response percentage to the baseline response percentage. With 20 quantiles, it is probable that 5% of the events occur in all quantiles. Thus, lift measures show how prospective is observing an event in each quantile compared to choosing random observations. The different values of lift measure for the different algorithms in train, validation, and test partitions are shown in Figure 4.

Sensitivity measure: the ROC curve is a graph of sensitivity against specificity grounded on the confusion matrix. These values are computed at different cut-off values. The Kolmogorov–Smirnov (KS) cut-off reference line is drawn at the value of 1-specificity for easing the identification of the most optimal cut-off to use while counting one's data, where the most significant variance between 1-specificity and sensitivity is detected for the VALIDATE partition.  Figure 5 shows the different values of sensitivity measures for the different algorithms in train, validation, and test partitions. The Kolmogorov–Smirnov statistic measures the distance between the reference distribution's cumulative distribution function and the sample's empirical distribution function or between the practical distribution functions of both models. In addition, when the K–S value gets lower than 0.05, one will learn that the lack of fit is significant.

Accuracy measure: accuracy is the observations' proportion, which is precisely categorized as an event or nonevent, and it is estimated at different cut-off values. Cut-off values range between 0 and 1, in increments of 0.05. At all cut-off values, the forecast target categorization is considered by if P_AttritionYes, the projected possibility of the event “Yes” for the target attrition, is bigger or equal to the cut-off value. When P_AttritionYes is bigger or equivalent to the cut-off value, then the predicted categorization is the event. Otherwise, it is a nonevent. Once the forecast categorization and the original classifications are both events (true positives) or nonevents (true negatives), the observation is rightly sorted. In case the expected sorting and real categorization contradict, then the observation is inaccurately sorted. The following is the formula to estimate accuracy.

(7) $$\begin{array}{c} \text{Acc.}=\;\frac{\text{true positive}+\text{true negative}}{\text{total obsrvations}}. \end{array}$$

Figure 6 shows the different values of accuracy measure for the different algorithms in train, validation, and test partitions.

F1 Score measure: the F1 score incorporates the criteria of precision and recall (or sensitivity), which are the measures of classification grounded on the confusion matrix estimated at different cut-off values. Cut-off values range between 0 and 1, in increments of 0.05. At all cut-off values, the forecast target categorization is considered by whether P_AttritionYes, the prophesied probability of the event “Yes” for the target attrition, is bigger or equal to the cut-off value. If P_AttritionYes is larger than or equivalent to the cut-off value, the foretold classification is an event. Otherwise, it is a nonevent.  Figure 7 shows the different values of the F1 score measure for the different algorithms in train, validation, and test partitions.

### 5.1. Models Fit Statistics Discussion

Tables 3–5 show differentfit statistic measuresthat are the basis for choosing the best or top model to be deployed in the production environments. Such measures are the Gini coefficient, misclassification rate, and average square error. The Gini coefficient is a statistic, measuring the degree of discrimination in a population. The Gini coefficient ranges between 0 and 1, where 0 represents perfect equivalence and 1 represents perfect discrimination [23]. Small Gini led to a better model, which is the gradient boosting in the test partition dataset. The misclassification rate is a performance metric, which informs the fraction of the wrong guesses without differentiating between negative and positive forecastings [24]. A low misclassification rate leads to a better model than others: the neural network model in the test dataset partition. There is no correct value for average square error (ASE). However, the lower the value, the better, and 0 means the model is perfect [25,26]. In our case, the better is the neural network model. A final word worth mentioning is that no model is better for all cases of businesses industries. However, we had selected the model that satisfies our analytics and business goals.

## 6. Conclusion and Future Work

The problem of maintaining good employees with experience threatens the owners of companies. The issue of employee attrition can cost employers a lot as it takes a lot to compensate for their expertise and efficiency. Hence, different machine learning techniques have been implemented with an ensemble model to find the different causes of such important business problems. Furthermore, multiple performance measures have been executed to discover the most effective machine learning techniques, such as cumulative lift, lift, accuracy, and F1 score. In addition, different models fit statistic measures were proposed. Such measures are the Gini coefficient, misclassification rate, and average square error that will be the basis for choosing the best or top model to be deployed in the production environments. The outcomes indicated that the lower value reflected the perfection of the model. However, findings revealed that no model up until now could be considered ideal and perfect for each case of business context. Yet, our chosen model was pretty much optimal as per our requirements and adequately satisfied the intended goal.

Lastly, it has been suggested that further studies should be conducted on the topic to contribute to a better understanding of the topic and present new outcomes supporting or opposing the current study and other literature available on this particular domain.

## Figures and Tables

**Figure 1:** Steps of the proposed model.

**Figure 2:** Mlp Neural Network.

**Figure 3:** Cumulative lift value for used algorithms.

**Figure 4:** Lift value for used algorithms.

**Figure 5:** Sensitivity value for used algorithms.

**Figure 6:** Accuracy value for used algorithms.

**Figure 7:** F1 score value for used algorithms.

**Algorithm 1:** Majority voting ensemble model.

**Table 1:** Overview of machine learning methods used for the prediction of employee turnover.

Ref.	Machine learning method										
	DT	RF	GBT	XGB	LR	SVM	NN	LDA	NB	KNN	AdaBoost
Alao and Adeyem	Yes	–	–	–	–	–	–	–	–	–	
Sisodia et al.	Yes	Yes				Yes			Yes	Yes	
Zhao et al.	Yes	Yes	Yes	Yes	Yes	Yes	Yes	Yes	Yes	Yes	
Yadav et al.	Yes	Yes			Yes	Yes					Yes
Alduayj, S. S. and Rajpoot, K. (2018)		Yes				Yes				Yes	
Falluchi et al.	Yes	Yes			Yes	Yes			Yes	Yes	

**Table 2:** Parameter values used in the preprocessing step.

Parameters	Parameter values
Maximum class level	20
Interval cut-off	20
Maximum missing percentage	50
Partitioning method	Stratify
Partitioning ratios	60 : 30 : 10
Imputation (missing values) method	Count for categorical variable
	Mean for interval variables

**Table 3:** Gini coefficient.

Partition	GB	NN	Forest	Ensemble
Train	−0.0335	0.6527	0.4671	0.5715
Validate	0.5078	0.7936	0.9826	0.8161
Test	0.3030	0.7704	0.6377	0.7326

**Table 4:** Misclassification rate.

Partition	GB	NN	Forest	Ensemble
Train	0.1633	0.1428	0.1701	0.1701
Validate	0.1609	0.1043	0.1088	0.1247
Test	0.1609	0.0861	0.1406	0.1337

**Table 5:** Average square error.

Partition	GB	NN	Forest	Ensemble
Train	0.138	0.10120	0.11953	0.113693
Validate	0.129	0.07701	0.06321	0.08596
Test	0.132	0.075362	0.107621	0.094548

## Data Availability

The data that support the findings of this paper are openly available at the SAS (www.sas.com) library.

## References

[1] Bhadoria R. S., Bhoj N., Zaini H. G. (2021). Artificial intelligence for creating low latency and predictive intrusion detection with security enhancement in power systems. *Applied Sciences*.

[2] Karthik S., Singh Bhadoria R., Gon Lee J. (2022). Prognostic kalman filter based bayesian learning model for data accuracy prediction. *Computers, Materials & Continua*.

[3] Jain P. K., Jain M., Pamula R. (2020). Explaining and predicting employees’ attrition: a machine learning approach. *SN Applied Sciences*.

[4] Chauhan S., Mittal M., Woźniak M., Gupta S., Pérez de Prado R. (2021). A technology acceptance model-based analytics for online mobile games using machine learning techniques. *Symmetry*.

[5] Sisodia D. S., Vishwakarma S., Pujahari A. Evaluation of machine learning models for employee churn prediction.

[6] Punnoose R., Ajit P. (2016). Prediction of employee turnover in organizations using machine learning algorithms. *International Journal of Advanced Research in Artificial Intelligence*.

[7] Alao D., Adeyemo A. B. (2013). Analyzing employee attrition using decision tree algorithms. *Computing, Information Systems, Development Informatics and Allied Research Journal*.

[8] Zhao Y. Employee turnover prediction with machine learning: a reliable approach.

[9] Yadav S., Jain A., Singh D. Early prediction of employee attrition using data mining techniques.

[10] Khare R., Kaloya D., Choudhary C. K., Gupta G. Employee Attrition risk assessment using logistic regression analysis.

[11] Alduayj S. S., Rajpoot K. Predicting employee attrition using machine learning.

[12] Zhu X., Seaver W., Sawhney R. (2017). Employee turnover forecasting for human resource management based on time series analysis. *Journal of Applied Statistics*.

[13] Fallucchi F., Coladangelo M., Giuliano R., William De Luca E. (2020). Predicting employee attrition using machine learning techniques. *Computers*.

[14] Jamalian E., Foukerdi R. (2018). A hybrid data mining method for customer churn prediction. *Engineering, Technology & Applied Science Research*.

[15] Arumugam A. (2017). A predictive modeling approach for improving paddy crop productivity using data mining techniques. *Turkish Journal of Electrical Engineering and Computer Sciences*.

[16] Elsalamony H. A. Detection of anaemia disease in human red blood cells using cell signature, neural networks and SVM. *Multimedia Tools and Applications*.

[17] Smitha N., Bharath R. Performance comparison of machine learning classifiers for fake news detection.

[18] Bhadoria R. S., Pandey M. K., Kundu P. (2021). RVFR: random vector forest regression model for integrated & enhanced approach in forest fires predictions. *Ecological Informatics*.

[19] Breiman L. (2001). Random forests. *Machine Learning*.

[20] Fernández-Delgado M., Cernadas E., Barro S., Amorium D. (2014). Do we need hundreds of classifiers to solve real world classification problems?. *Journal of Machine Learning Research*.

[21] Bentéjac C., Csörgő A., Martínez-Muñoz G. (2021). A comparative analysis of gradient boosting algorithms. *Artificial Intelligence Review*.

[22] Friedman J. H. (2001). Greedy function approximation: a gradient boosting machine. *Annals of Statistics*.

[23] Dorfman R. (1979). A formula for the Gini coefficient. *The Review of Economics and Statistics*.

[24] Aoshima M., Yata K. (2014). A distance-based, misclassification rate adjusted classifier for multiclass, high-dimensional data. *Annals of the Institute of Statistical Mathematics*.

[25] Barron A. R. (1984). Predicted squared error: a criterion for automatic model selection. *Self-organizing methods in modeling GMDH type algorithms*.

[26] Ounpraseuth S., Lensing S. Y., Spencer H. J., Kodell R. L. (2012). Estimating misclassification error: a closer look at cross-validation based methods. *BMC Research Notes*.

